This article has been retracted.

# Possible Role of Interaction between PPAR*α* and Cyclophilin D in Cardioprotection of AMPK against* In Vivo* Ischemia-Reperfusion in Rats

**DOI:** 10.1155/2016/9282087

**Published:** 2016-03-08

**Authors:** Giselle Barreto-Torres, Sabzali Javadov

**Affiliations:** Department of Physiology, University of Puerto Rico School of Medicine, San Juan, PR 00936-5067, USA

## Abstract

Activated AMPK protects the heart from cardiac ischemia-reperfusion (IR) injury and is associated with inhibition of mitochondrial permeability transition pore (PTP) opening. On the other hand, pharmacological inhibition of the PTP reduces infarct size and improves cardiac function. However, it is unclear whether beneficial effects of AMPK are mediated through the PTP and, if they are not, whether simultaneous activation of AMPK and inhibition of the PTP exert synergistic protective effects against cardiac IR injury. Here, we examined the effects of the AMPK activator, A-769662 in combination with the PTP inhibitor, sanglifehrin A (SfA) on* in vivo* cardiac IR. Cardiac dysfunction following IR injury was associated with decreased activity of the mitochondrial electron transport chain (ETC) and increased mitochondrial ROS and PTP opening. Administration of A-769662 or SfA individually upon reperfusion improved cardiac function, reduced infarction size, and inhibited ROS production and PTP opening. However, simultaneous administration of SfA and A-769662 did not provide synergistic improvement of postischemic recovery of cardiac and mitochondrial function, though both compounds disrupted IR-induced interaction between PPAR*α* and CyP-D. In conclusion, A-769662 or SfA prevents PPAR*α* interaction with CyP-D, improving cardiac outcomes and increasing mitochondrial function, and simultaneous administration of the drugs does not provide synergistic effects.

## 1. Introduction 

AMPK is a serine/threonine kinase that is activated by increased intracellular AMP levels. In the heart, AMPK has been shown to regulate cellular uptake and subsequent entry of fatty acids into the mitochondria to increase fatty acid oxidation [1]. Also, AMPK stimulates translocation of GLUT-4 to the sarcolemma to increase glucose uptake [2] and activates glycolysis [3]. AMPK is activated in response to oxidative and energy stress induced by ischemia-reperfusion (IR) in the heart [4, 5]. Notably, increased AMP/ATP ratio in cardiac IR activates AMPK through stimulation of threonine (Thr^172^) phosphorylation [4] or inhibition of AMPK dephosphorylation [5]. Active AMPK switches off energy-consuming processes like protein and lipid synthesis and stimulates ATP-generating mechanisms thereby maintaining ATP production despite the lack of oxygen in the heart [6–8]. Previous studies using genetic mouse models lacking the cardiac-specific *α*2-AMPK isoform have collectively demonstrated that downregulation of AMPK induces greater cardiac injury, activates apoptosis, and worsens cardiac recovery after IR [9, 10], whereas the activation of AMPK protects the heart and improves mitochondrial function [11].

Based on the potential therapeutic benefits observed in animal models, extensive studies have been performed to develop pharmacological activators of AMPK. Early studies determined that biguanides, including metformin, increased the phosphorylation and activation of AMPK, thereby protecting the heart against IR injury [12]. Yet, the mechanism of metformin in AMPK activation is still poorly understood. Metformin has been shown to exert pleiotropic effects, activating AMPK-independent pathways of cell survival [13]. Also, numerous studies suggest that metformin acts through the inhibition of the electron transport chain (ETC) complex I, increasing AMP levels due to inhibition of oxidative phosphorylation [14, 15]. Notably, the inhibition of AMPK activity prevented the cardioprotective effects of metformin, suggesting a central role of AMPK in mediating beneficial effects of metformin. Furthermore, the beneficial effects of metformin are abrogated by inhibition of the p38 mitogen-activated protein kinase and PKC [13]. Interest in the development of a more specific AMPK activator led to the identification of a potent thienopyridone called A-769662. Instead of activating AMPK indirectly by increasing the AMP : ATP ratio, A-769662 directly binds to the regulatory *β*-subunit of AMPK and, thereby, allosterically stimulates AMPK [16]. A-769662 has also been shown to inhibit AMPK dephosphorylation and increase AMPK resistance to protein phosphatases [17].

The cardioprotective effects of AMPK activation are associated with inhibition of the mitochondrial permeability transition pores (PTP) [18–20]. The PTP is a nonselective channel that renders mitochondria permeable to any solute up to approximately 1.5 kDa, inducing mitochondrial swelling. In turn, the outer membrane ruptures, releasing proapoptotic factors that eventually stimulate cell death via apoptosis or necrosis [21, 22]. Although the molecular identity of the PTP complex is controversial, a key regulator of the pores is cyclophilin D (CyP-D), a cis-trans isomerase found exclusively in the mitochondrial matrix that is essential for proper protein folding [23].

In this study, we examined whether simultaneous PTP inhibition and AMPK activation provided synergistic cardioprotection against* in vivo* cardiac IR. To avoid the undesired AMPK-independent effects of metformin, we used A-769662 in this study to activate AMPK. Since AMPK mediates cardioprotection by inhibiting PTP opening, we hypothesized that combined treatment with SfA and A-769662 would not provide synergistic effects. Our experiments revealed that treatment with SfA and/or A-769662 protects cardiac function and mitochondria without affecting AMPK phosphorylation. Both individual treatments reduced mitochondrial ROS (mitROS) levels, improved the activities of ETC complexes, and prevented IR-induced PPAR*α*-CyP-D interaction and PTP opening. The combination of SfA and A-769662 did not provide synergistic cardioprotective effects on cardiac IR.

## 2. Materials and Methods

### 2.1. Animals

Male Sprague-Dawley rats (250–275 g, Charles River, Wilmington, MA) were housed in individual cages in a temperature controlled room under a regular light-dark cycle. Water and food were provided* ad libitum*. All experiments were performed according to protocols approved by the University Animal Care and Use Committee and conformed to the National Research Council Guide for the Care and Use of Laboratory Animals published by the US National Institutes of Health (2011, eighth edition).

### 2.2. *In Vivo* Model of Cardiac IR

Animals were anesthetized with an anesthetic cocktail containing (mg per kg body weight, IP) xylazine 4.2, ketamine 87.5, and acepromazine 0.88 and artificially ventilated with room air using a small-animal ventilator (Kent Scientific Corp., Torrington, CT). The respiration rate was maintained at 65 to 70 breaths per minute, and body temperature was maintained at 37°C by placing the animals on a homeothermic surgery table [24]. Lateral thoracotomies were performed to gently expose the hearts. The left anterior descending coronary arteries were ligated ~3 mm from their origins with firmly tied silk sutures (7-0), inducing myocardial infarction. Electrocardiograms (ECG) were recorded to monitor the hearts' electrical activity throughout the surgeries by using the MouseMonitor*™* (Indus Instruments, Houston, TX) heating pad with needle ECG leads. For the Sham procedures the ligatures were placed in an identical fashion but not tied. The resulting coronary artery ligations (CAL) were maintained for 30 min, after which the sutures were removed and followed by reperfusion for 24 h. The animals were randomly divided into the following five groups: Sham (no CAL, *n* = 7), IR (*n* = 8), IR + SfA (*n* = 4), IR + A-769662 (IR + A, *n* = 6), and IR + SfA + A-769662 (IR + SfA + A, *n* = 4). Animals having no ST-segment elevation on the ECG following CAL were excluded from IR groups with or without treatment due to a lack of myocardial infarction. SfA (25 mg/kg), A-769662 (10 mg/kg), or their combination was administered by intravenous bolus immediately before reperfusion. The doses for SfA and A-769662 were based on previous studies that demonstrated that SfA treatment [25] or A-769662 treatment [26] had cardioprotective effects in murine models of* in vivo* IR.

### 2.3. Echocardiography

Echocardiographic measurements were performed as described previously [24]. Briefly, rats were anesthetized and placed in a supine position. M-mode and 2D echocardiography images were obtained with a high-frequency 8–4 MHz 10-mm broadband phased P10 probe attached to a digital portable ultrasound system Micromaxx (Sonosite Inc., Bothell, WA). Diastolic and systolic measurements of LV dimensions (LVIDd, LVIDs), LV end-systolic and end-diastolic volumes (LVESV, LVEDV), and HR were recorded. Then, stroke volume (SV), cardiac output (CO), and ejection fraction (EF) were calculated as SV = LVEDV − LVESV, CO = (SV*∗*HR)/1000, and EF = ((LVEDV − LVESV)/LVEDV)*∗*100, respectively.

### 2.4. Infarction Size

Rats were sacrificed, the hearts were excised, and blood was washed for 10 min by retrograde perfusion with Krebs-Henseleit solution [27]. Then, the hearts were placed in −20°C for 1-2 h, manually sliced into 5-6 uniform slices, and incubated for 20 min in the phosphate buffer (0.1 M Na_2_HPO_4_ and 0.1 M NaH_2_PO_4_, pH 7.4 at 37°C) containing 10 mg/mL tetrazolium chloride (TTC). The heart sections were fixed in 10% formaldehyde overnight and then photographed. Digital images of heart sections were analyzed for infarct size (TTC negative) using the NIH ImageJ software. The infarction size was calculated as a percentage of the entire left ventricle.

### 2.5. Measurement of PTP Opening in Isolated Mitochondria

Opening of the mitochondrial pore was determined by Ca^2+^ induced swelling of isolated mitochondria, measured as a reduction in light scattering at 520 nm, as previously described [28]. Mitochondria containing 50 *μ*g of protein were incubated at 25°C in 200 *μ*L buffer containing 150 mM KSCN, 20 mM MOPS, 10 mM Tris, and 2 mM nitrilotriacetic acid, supplemented with 0.5 *μ*M rotenone, 0.5 *μ*M antimycin, and 2 *μ*M A23187. Swelling of mitochondria was initiated by progressive additions of CaCl_2_ (100 *μ*M every 5 min for a total of 5 times), and rates of swelling were determined by monitoring the decrease in light scattering at 525 nm, quantified using a Spectramax M3 plate reader (Molecular Devices, Sunnyvale, CA, USA).

### 2.6. Mitochondrial ETC Complexes Enzyme Activity

Enzymatic activities of ETC complexes were determined in isolated cardiac mitochondria, as previously described [29]. Briefly, mitochondria were diluted with a hypertonic media buffer (25 mM KH_2_PO_4_, 5 mM MgCl_2_, and 0.5 mg/mL BSA), supplemented with saponin (0.55 mg/mL). To access the ETC complexes embedded in the inner mitochondrial membrane, the mitochondria were disrupted three times by freeze-thawing and, then, incubated for 30 min at 4°C. All measurements were recorded at the Thermo Scientific GENESYS*™* 10S UV-Vis spectrophotometer at 30°C. Activities of all ETC complexes were normalized to citrate synthase activity.

*Citrate synthase activity* was determined by measuring coenzyme A formation at the Thermo Scientific GENESYS*™* 10S UV-Vis spectrophotometer and was expressed as nmol oxaloacetate/min per mg protein [28].

### 2.7. Mitochondrial ROS Levels

Amplex Red (Life Technologies, Carlsbad, CA), a dye that reacts with H_2_O_2_ to produce the highly fluorescent molecule, resorufin, was used for measurement of ROS levels in isolated mitochondria. Mitochondria were incubated with 100 *μ*M Amplex Red for 15 min, and the fluorescence intensity was quantified using a Spectramax M3 plate reader (Molecular Devices, Sunnyvale, CA, USA) at an excitation of 460 nm and emission of 490 nm.

### 2.8. SDS-PAGE and Western Blotting

Protein concentration in homogenate and mitochondria was determined by the Bradford assay (Bio-Rad, Hercules, CA). Equal amounts (50 *μ*g/well) of protein were loaded onto 10% SDS-PAGE gels, run, and transferred onto Amersham Hybond ECL nitrocellulose membranes (GE Healthcare Bio-Sciences Corp., Piscataway, NJ). The membranes were immunoblotted with AMPK, P-AMPK*α*_1_^Thr172^ (Cell Signaling, Boston, MA), PPAR*α*, and P-PPAR*α* ^Ser21^ (Santa Cruz Biotechnology, Santa Cruz, CA). The signals were visualized using Thermo Scientific Pierce ECL Western Blotting Detection reagents (Thermo Scientific, Rockford, IL) at the VersaDoc 3000 Gel Imaging System (Bio-Rad, Hercules, CA).

### 2.9. Co-Immunoprecipitation

Protein samples were incubated with anti-PPAR*α* or anti-CyP-D antibodies overnight at 4°C, and the immunoprecipitates were harvested with Dynabeads® Protein G (Life Technologies, Carlsbad, CA). The immunoprecipitated complexes were washed and, then, subjected to SDS-PAGE, followed by immunoblotting using antibodies for CyP-D (Abcam, Cambridge, MA) or PPAR*α*.

### 2.10. Statistical Analysis

Data are presented as means ± SE. Differences among groups were compared by two-tailed Student's* t*-tests. Differences were considered to be statistically significant when *P* < 0.05.

## 3. Results

### 3.1. Cardiac Function and Infarct Size

The heart-to-body weight ratio (HW/BW) was increased by 24% (*P* < 0.05) in the IR group compared to Sham-operated rats. Treatment with A-769662 and/or SfA significantly prevented the IR-induced increase of the HW/BW ratio (Figure 1(a)).

Next, we determined the effects of A-769662 and/or SfA on infarct size with the TTC method. As shown in Figures 1(b) and 1(c), the infarct size was 71% (*P* < 0.01), 33% (*P* < 0.05), and 49% (*P* < 0.05) less in IR + A-769662, IR + SfA, and IR + SfA + A groups, respectively, compared to the IR group. Interestingly, SfA alone did not reduce infarct size as much as the other two treatments (A-769662 and SfA + A-769662). Analysis of cardiac function demonstrated that rats subjected to IR had a 51% and 55% (*P* < 0.01 for both) lower cardiac output and ejection fraction, respectively, than the Sham-operated counterparts (Figures 2(a) and 2(b)). In all treatment groups, cardiac output and ejection fraction were remarkably preserved compared to the IR (untreated) group. No significant differences were observed between the treated groups with regard to changes of cardiac output and ejection fraction.

Overall, these results suggest that activation of AMPK and inhibition of PTP protect the heart during cardiac IR by reducing infarct size and improving cardiac function.

### 3.2. Phosphorylation of AMPK and PPAR*α*

We examined the effects of A-769662 and/or SfA on phosphorylation of AMPK and PPAR*α* during cardiac IR. Results demonstrated a 2-fold (*P* < 0.05 versus Sham) increase in P-AMPK^Thr172^ levels in IR hearts. Neither treatment with A-769662 nor treatment with SfA had any effects on IR-induced AMPK phosphorylation. However, simultaneous treatment with SfA and A-769662 returned the expression of P-AMPK^Thr172^ to the level shown in Sham-operated hearts (Figures 3(a) and 3(b)). Also, IR, with or without treatment, increased the level of P-PPAR*α* by 100%, 88%, 68%, and 68% (*P* < 0.05 for all) in IR, IR + A-769662, IR + SfA, and IR + SfA + A, respectively, compared to the Sham group (Figures 3(d) and 3(e)). Total levels of AMPK and PPAR*α* were not affected by IR, with or without treatment (Figures 3(c) and 3(f)).

Overall, these results indicate that, unlike metformin, A-769662 does not phosphorylate AMPK at Thr^172^. Furthermore, cardiac IR-stimulated PPAR*α* phosphorylation is not prevented by A-769662 and/or SfA.

### 3.3. Mitochondrial PTP Opening and mitROS Production

In the next set of experiments, we evaluated the effects of A-769662, SfA, or the combination on mitROS production in cardiac IR. We measured H_2_O_2_ levels in isolated mitochondria using the Amplex Red assay. IR induced a 54% (*P* < 0.01) increase of mitROS levels compared to the Sham group, and treatment with A-769662 and/or SfA at reperfusion blocked the IR-induced increase of mitROS levels (Figure 4(a)). Since elevated mitROS levels play a causal role in cell damage by inducing PTP opening, we assessed whether pore opening is affected by cardiac IR, with or without treatment. As shown in Figures 4(b) and 4(c), hearts subjected to IR had an 80% (*P* < 0.01 versus Sham) increase in Ca^2+^-induced mitochondrial swelling (a marker of PTP opening), which was significantly attenuated in all three treatment groups (IR + A-769662, IR + SfA, and IR + SfA + A-769662). Altogether, these data demonstrate that treatment with A-769662 and/or SfA decreases mitROS levels and inhibits PTP opening.

### 3.4. Enzymatic Activity of Mitochondrial ETC Complexes

Analysis of enzymatic activity of ETC complexes demonstrated that cardiac IR reduced the activity of complexes I, III, and IV by 28%, 44%, and 50% (*P* < 0.05 for all), respectively, compared to Sham-operated animals (Figure 5). Treatment with A-769662 improved the activities of complexes I and IV, which were 23% and 40% (*P* < 0.05) higher, respectively, compared to the IR group. Likewise, the activities of complexes I and IV in SfA-treated hearts were 38% and 47% (*P* < 0.05 for both) higher, respectively, than that in untreated hearts. The combination of SfA with A-769662 did not exert additional effects on the activity of the ETC complexes. Likewise, neither treatment with SfA, A-769662 nor the combination improved IR-induced suppression of complex III activity (Figure 5(b)).

Next, we measured citrate synthase activity as a marker of mitochondrial mass. Our results showed that IR reduced citrate synthase activity in mitochondria. Treatment with SfA, A-769662, or their combination did not prevent the effect of IR, suggesting that improvements observed with ETC complexes are not due to increased mitochondrial mass (Figure 5(d)).

These results demonstrate that cardiac IR decreased the activity of ETC complexes I, II, III, and IV. Furthermore, A-769662 and/or SfA significantly prevented inactivation of all the complexes, except for complex III.

### 3.5. Physical Interaction between CyP-D and PPAR*α*

In our* in vitro *studies, oxidative stress stimulated protein-protein interactions between PPAR*α* and CyP-D in H9c2 cardioblasts, and those interactions were prevented by metformin [20]. Therefore, we sought to examine whether PPAR*α* and CyP-D interaction occurred in an* in vivo* model of cardiac IR. We applied two contrasting technical approaches to verify the interaction when mitochondrial proteins were immunoprecipitated with PPAR*α* or CyP-D antibodies followed by immunoblotting with CyP-D or PPAR*α* antibodies (Figures 6(a) and 6(b)). In both cases, cardiac IR significantly increased interactions between PPAR*α* and the PTP regulator, CyP-D (*P* < 0.05), when compared with the Sham group. However, treatment with A-769662 and/or SfA ameliorated this interaction (Figures 6(a) and 6(b)). In conclusion, these data demonstrate the existence of physical interactions between PPAR*α* and CyP-D in response to IR, and A-769662 and/or SfA are able to abrogate these interactions.

## 4. Discussion 

This study demonstrated that (i) SfA, A-769662, or their combination attenuated cardiac dysfunction and infarct size induced by* in vivo* IR; (ii)* in vivo* cardiac IR increased phosphorylation of AMPK, which was not affected by treatments with A-769662; (iii) SfA, A-769662, or their combination reduced IR-induced mitROS levels and PTP opening in cardiac mitochondria; (iv)* in vivo* cardiac IR induced an interaction between PPAR*α* and CyP-D which was attenuated by SfA, A-769662, or their combination; and (v) IR-induced decrease in ETC activity was abrogated by SfA, A-769662, or their combination. These data, for the first time, provide evidence that although both AMPK activation and PTP opening exert cardioprotective effects against* in vivo* IR, the simultaneous application of both therapeutic approaches (SfA + A-769662) has no synergistic effects.

Activation of AMPK by A-769662 has been previously shown to protect endothelial [30], neuronal [31], and liver [32] cells, as well as the whole heart [26, 33], from oxidative damage. A-769662 protected hearts against IR injury, and this protection was associated with decreased infarct size and PTP opening in Goto-Kakizaki diabetic rats [18]. However, there are no studies elucidating simultaneous effects of AMPK activation and PTP inhibition on cardiac IR. Our results show that A-769662 and SfA independently protected hearts against cardiac IR, as evidenced by reduced infarct size and improved cardiac output and ejection fraction. Interestingly, the protective effects provided by combined therapy of A-769662 and SfA on infarct size and cardiac function were similar to those provided by A-769662 alone. Based only on these data, it is impossible to conclude whether these compounds had synergistic or nonsynergistic effects. Interestingly, SfA treatment alone did not reduce infarct size as much as A-769662, although it protected cardiac function as much as A-769662 or A-769662 + SfA. These results suggest that the cardioprotective mechanism of PTP inhibition is not dependent solely on infarct size reduction, but rather due to additional beneficial effects such as coronary vasodilation. Another possible explanation for these findings is that A-769662 could also activate other PTP-independent mechanisms to decrease infarct size.

Previous studies found that pretreatment with A-769662 did not stimulate phosphorylation of AMPK at Thr^172^ in the Langendorff-perfused mouse heart subjected to* ex vivo* IR [26]. However, treatment with A-769662 in combination with other classical AMPK activators (metformin, AICAR, phenformin, and oligomycin) induced a dramatic increase in AMPK phosphorylation and stimulated glucose uptake [34]. It has been suggested that A-769662 activates AMPK by not increasing its phosphorylation at the Thr^172^ site of the alpha subunit; it acts through the regulatory *β*-subunit to allosterically activate AMPK and its downstream targets [26]. Consistent with this, we observed no further increase in P-AMPK^Thr172^ levels in the hearts pretreated with A-769662.

It has been suggested that the cardioprotective effects of AMPK activation are mediated mainly through the mitochondria. Mitochondria isolated from mouse hearts expressing kinase-dead (KD) AMPK demonstrated increased hydrogen peroxide production and decreased resistance to PTP opening compared to WT counterparts [35]. Conversely, pretreatment with A-769662 inhibited PTP formation, induced by* ex vivo *IR, in Langendorff-perfused hearts [18] and oxidative stress in H9c2 cardioblasts [20]. Consistent with these studies, we found that A-769662 causes inhibition of the PTP immediately upon reperfusion in* in vivo* cardiac IR. CyP-D is a key regulator of the PTP and has emerged as an important target for PTP inhibition [21, 36]. The pharmacological inhibitors of CyP-D, CsA, and SfA, have been shown to attenuate PTP opening and exert cardioprotective effects against IR [25, 37–39]. SfA is a CsA analogue that, unlike CsA, does not inhibit the activity of the Ca^2+^-activated phosphatase, calcineurin [37]. Furthermore, SfA and CsA inhibit PTP opening through different mechanisms; CsA prevents interaction of CyP-D with the adenine nucleotide translocase, another key PTP regulator, whereas SfA inhibits the enzymatic activity of CyP-D [36].

Notably, PTP opening occurs at reperfusion, but not during ischemia, and reaches a maximum within 10–15 min of reperfusion [36, 40]. Cardioprotective effects were observed only when SfA was administered during the first 15 min of reperfusion. Administration of SfA after 15 min of reperfusion had no cardioprotection against* ex vivo* IR injury [39]. Likewise, SfA administered 5 min prior to reperfusion showed a marked decrease in infarct size [25]. In line with these studies, in our experiments, SfA was administered immediately upon reperfusion, which significantly abrogated cardiac dysfunction and reduced infarct size. Choosing the right time to administer PTP inhibitors is apparently important for maximum protective effects in treatment of cardiac IR. This factor might be one of the main reasons that the recent CIRCUS clinical trials with CsA failed to protect hearts against reperfusion injury in STEMI patients [41].

Although we and others have established that the beneficial effects of AMPK activation against cardiac IR are mediated through PTP formation, the specific mechanisms associated with AMPK-induced inhibition of the PTP are still unclear. One potential mechanism may involve the indirect modulation of CyP-D. We have previously shown that the beneficial effects of metformin on mitochondria are mediated through PPAR*α*, since the PPAR*α* inhibitor GW6471 prevented cardioprotective effects of metformin against IR in rat hearts [19]. PPAR*α* is one of central mediators involved in the mitochondrial transcriptional network that regulates cardiac mitochondrial metabolism and biogenesis under both physiological and pathological conditions [42, 43]. PPAR*α* seems to be a downstream target for AMPK that could modulate PTP formation. Indeed, our studies with cultured H9c2 cells demonstrated that H_2_O_2_-induced oxidative stress promoted protein-protein interactions between PPAR*α* and CyP-D that were associated with PTP opening. Conversely, activation of AMPK prevented this interaction, suggesting that AMPK was indirectly involved in regulating pore formation by diminishing the interaction of PPAR*α* with CyP-D [20]. Likewise,* in vivo* cardiac IR induces protein-protein interactions between PPAR*α* and CyP-D (Figure 6), and pretreatment with A-769662 abrogated this interaction, confirming the results previously observed with our* in vitro *model of oxidative stress.

Our data also indicate that the mechanism underlying the protective action of A-769662 is not associated with phosphorylation of PPAR*α*. Inhibition of the PTP might be due to phosphorylation of GSK-3*β*, a downstream target of AMPK activation. Recent studies demonstrate that A-769662 increased the phosphorylation of GSK-3*β*, inhibiting PTP formation [18] and reducing the levels of mitROS [44] in cardiac IR. AMPK could also inhibit the PTP through posttranslational modifications of CyP-D. Previous studies have demonstrated that acetylation of CyP-D [24, 45] can also initiate its interaction with other proteins and promote PTP formation. We have showed that the beneficial effects of metformin against oxidative stress-induced injury were not associated with acetylation or phosphorylation of CyP-D, although other types of posttranslational protein modifications may be involved [23]. Recent studies demonstrated a possible role of AMPK-induced JNK inhibition to increase the resistance of cardiac mitochondria to PTP opening in the kinase-dead AMPK mouse [35]. However, in our previous studies, the specific JNK inhibitor SU3327 had noninhibitory effects on the mitochondrial PTP in rat hearts subjected to global IR [28].

In summary, combination of A-769662 and SfA exerted no additional protective effects on cardiac function, mitochondrial ETC activity, PTP opening, or mitROS levels compared to individual treatments. On the other hand, it is difficult to make conclusion on the synergistic effect of A-769662 and SfA as treatment with each compound returned the changes observed in IR to the Sham level for most parameters. Further studies are needed to elucidate the synergistic effect of AMPK activation and PTP inhibition and understand the molecular mechanisms of cardioprotection induced by the AMPK/PTP pathway.

## Figures and Tables

**Figure 1:** Effects of A-769662 (A) and/or SfA on the heart-to-body weight ratio (HW/BW) and infarct size during cardiac IR. (a) HW/BW expressed as a fold change of the Sham group; (b) representative images of heart cross sections, showing viable (*red*) and infarcted tissue (*white*) for all experimental groups; (c) quantitative results of TTC staining, expressed as percentages of the IR group. The number of animals in each group for analysis of HW/BW (a): Sham (*n* = 7), IR (*n* = 8), IR + SfA (*n* = 4), IR + A-769662 (*n* = 6), and IR + SfA + A (*n* = 4). Additional 3 hearts from each group were analyzed for quantification of infarction size (b and c). ^*∗*^ *P* < 0.01 versus Sham; ^#^ *P* < 0.05, ^##^ *P* < 0.01 versus IR; ^+^ *P* < 0.01 versus IR + A and IR + SfA + A.

**Figure 2:** Effects of A-769662 (A) and/or SfA on cardiac output (a) and ejection fraction (b) of hearts after IR or Sham procedure. Calculations of cardiac output and ejection fraction are given in Section 2. The number of animals: Sham (*n* = 7), IR (*n* = 8), IR + SfA (*n* = 4), IR + A-769662 (*n* = 6), and IR + SfA + A (*n* = 4). ^*∗*^ *P* < 0.01 versus Sham; ^#^ *P* < 0.01 versus IR.

**Figure 3:** Protein levels of phosphorylated and total AMPK*α* (a–c) and PPAR*α* (d–f) in heart homogenates. Protein levels of P-AMPK*α*_1_^Thr172^ and P-PPAR*α* ^Ser21^ were normalized to total AMPK*α*_1_ and PPAR*α*, respectively, whereas the levels of AMPK and PPAR*α* were normalized to GAPDH. Top panels (a, d) are representative western blots in each group. Bottom panels represent quantitative data of protein expression for P-AMPK*α*_1_^Thr172^ (b), AMPK*α*_1_ (c), P-PPAR*α* ^Ser21^ (e), and PPAR*α* (f). Results are expressed as a fold change of the Sham group. The number of animals: Sham (*n* = 7), IR (*n* = 8), IR + SfA (*n* = 4), IR + A-769662 (*n* = 6), and IR + SfA + A (*n* = 4). ^*∗*^ *P* < 0.05 versus Sham; ^#^ *P* < 0.05 versus IR.

**Figure 4:** ROS levels and Ca^2+^-induced mitochondrial swelling as an indicator of PTP opening in cardiac mitochondria isolated from rats treated with A-769662 (A) and/or SfA. (a) ROS levels in mitochondria, expressed as pmoles of H_2_O_2_ per mg of protein per minute. (b) Representative traces of mitochondrial swelling, shown as calcium-induced decrease in light scattering at 520 nm. (c) Quantitative data of PTP opening, shown as the rate of swelling and expressed in percentage of maximum swelling induced by 0.5 mM CaCl_2_. The number of animals: Sham (*n* = 7), IR (*n* = 8), IR + SfA (*n* = 4), IR + A-769662 (*n* = 6), and IR + SfA + A (*n* = 4). ^*∗*^ *P* < 0.01 versus Sham; ^#^ *P* < 0.01 versus IR.

**Figure 5:** Effects of SfA, A-769662 or their combination (A) on the activity of the ETC complexes I (a), III (b), and IV (c), and citrate synthase (d) in cardiac mitochondria. Activities of ETC complexes and citrate synthase (CS) were normalized to citrate synthase or mg mitochondrial protein, respectively. ^#^ *P* < 0.05, ^##^ *P* < 0.01 versus IR, ^*∗*^ *P* < 0.05, ^*∗∗*^ *P* < 0.01 versus Sham.

**Figure 6:** Effects of SfA, A-769662, or their combination on IR-induced CyP-D-PPAR*α* interaction. Isolated mitochondria were immunoprecipitated (IP) with anti-PPAR*α* (a) or anti-CyP-D (b) antibodies. The complexes were subjected to SDS-PAGE, followed by immunoblotting (IB) with CyP-D (a) or PPAR*α* (b) antibodies. Representative immunoblots (a and b, top panels) show the effects of A-769662 and/or SfA on the interaction between PPAR*α* and CyP-D. Quantitative results (a and b, bottom panels) were expressed as a fold change, compared with Sham. *n* = 3-4 per each group. ^*∗*^ *P* < 0.05 versus Sham; ^#^ *P* < 0.05 versus IR.

## Abbreviations

AMPK: AMP-activated protein kinase
CsA: Cyclosporin A
CyP-D: Cyclophilin D
ECG: Electrocardiography
ETC: Electron transport chain
IR: Ischemia-reperfusion
HW/BW: Heart weight to body weight ratio
CAL: Coronary artery ligation
mitROS: Mitochondrial ROS
PGC-1*α*: PPAR-gamma co-activator 1-alpha
PPAR: Peroxisome proliferator-activated receptor
PTP: Permeability transition pore
ROS: Reactive oxygen species
SfA: Sanglifehrin A
TTC: 2,3,5-Triphenyltetrazolium chloride.
